# Development and Performance Verification of a Motorized Prosthetic Leg for Stair Walking

**DOI:** 10.1155/2020/8872362

**Published:** 2020-10-27

**Authors:** Kiwon Park, Hyoung-Jong Ahn, Kwang-Hee Lee, Chul-Hee Lee

**Affiliations:** ^1^Department of Mechatronics Engineering, Incheon National University, Incheon 22012, Republic of Korea; ^2^Department of Mechanical Engineering, Inha University, Incheon 22212, Republic of Korea

## Abstract

The present study emphasized on the optimal design of a motorized prosthetic leg and evaluation of its performance for stair walking. Developed prosthetic leg includes two degrees of freedom on the knee and ankle joint designed using a virtual product development process for better stair walking. The DC motor system was introduced to imitate gait motion in the knee joint, and a spring system was applied at the ankle joint to create torque and flexion angle. To design better motorized prosthetic leg, unnecessary mass was eliminated via a topology optimization process under a complex walking condition in a boundary considered condition and aluminum alloy for lower limb and plastic nylon through 3D printing foot which were used. The structural safety of a developed prosthetic leg was validated via finite element analysis under a variety of walking conditions. In conclusion, the motorized prosthetic leg was optimally designed while maintaining structural safety under boundary conditions based on the human walking data, and its knee motions were synchronized with normal human gait via a PD controller. The results from this study about powered transfemoral prosthesis might help amputees in their rehabilitation process. Furthermore, this research can be applied to the area of biped robots that try to mimic human motion.

## 1. Introduction

A prosthetic leg is a basic rehabilitation device that helps rehabilitation of limb amputees, and the number of lower-limb amputees was estimated at approximately 7 million worldwide [1]. The development of prosthetic legs for lower-limb amputees is becoming an important issue. The above-knee amputees and particularly the lower-limb amputees' face increased difficulties in natural walking when compared with lower-knee amputees. This is because of the absence of the knee joints that are mainly responsible (50% of the importance) for the walking mechanism. The development of prosthetic leg that can create the natural knee motion is required for above-knee amputees.

The prosthetic leg can be classified as passive, variable-damping, or powered [2–4]. Prosthetic legs were traditionally classified as passive or variable-damping due to limitations of power generation and battery life. Passive and variable-damping types do not result in a natural motion in keeping with user intentions. Hence, the powered type is considered to replace the passive and variable-damping types. Powered prosthetic legs are enabled by advances in computers, robotics, and battery technology [5]. Powered prosthetic legs can be classified based on their method of torque generation as three linkage types or direct-drive types. Conventional three linkage types are an easy way to convert the linear motion to the rotating motion at the knee joint. However, a longer linkage is required to generate a large angle at the knee joint due to kinematics and leads to issues with the dimensions. Additionally, the center of mass shifts when the translation linkage shortens. The direct-drive type directly transfers the rotational motion of the motor to the joint. However, it requires an additional device to amplify the torque, which can increase the size and weight of the prosthesis.

There have been different kinds of studies about the development of powered prosthetic leg. Some researcher used electrohydraulic actuator for making the knee motion [6]. Due to advances in motor and battery technology, the motor is introduced as an actuator of a prosthetic leg. Three linkage type powered prosthetic leg was developed using a motor and ball screw system [7, 8]. As motors become more compact and are enable to produce high torque, direct-drive type prostheses have been developed. DC motor was used for the drive system [9–11] or a harmonic drive and belt pulley system to amplify the torque applied to the knee joint [12]. Studies were performed on the kinematic structure design of an active prosthetic leg with a motor system [13, 14]. The extant research examined control mechanisms of knee and ankle joints to mimic a natural human gait [15, 16]. However, most previous studies focused on the kinematic walking mechanism or control for the level walking. Only a few studies carried out for control mechanisms under stair walking condition [9].

Most of the study of the powered prosthetic leg focused on overground walking, but for the disabled to move freely, a prosthetics capable of overcoming various obstacles should be developed. Typical walking obstacles include ramps and stairs, of which obstacles requiring greater power are stairs. In order to climb the stairs, it should be considered for various dynamic loads and requires more power than when walking on the overground. Therefore, it is inevitably required to be lightweight and an optimum structure that is as stable as possible under limited weight conditions. Existing studies focus on control to overcome the staircase, and research on optimizing the structure itself is insufficient. The purpose of this study was to perform the optimization of a motorized prosthesis capable of walking on stairs.

Several major factors influence the behavior of a prosthetic leg and include the alignment, mechanical properties, length, and the weight of the components of a prosthetic leg [17]. Although the weight of the prosthesis is one of the important factors for performance, researches to improve the structure of the prosthesis are rarely carried out. In order to overcome obstacles such as stair, it is necessary to study the optimization of the structure of prosthetic legs. Recently, studies about a prosthetic leg for walking stairs have been actively carried out, but little research has been implemented to design optimal structures for stair walking.

This study focuses on the development of a powered transfemoral prosthetic leg that can imitate the human walking motion and is optimized for stair walking. A structural design with two degrees of freedom at the knee and ankle joint was proposed. The power system of the knee joint is most important because the knee joint plays a major role (exceeding 50%) in the walking mechanism. In order to produce a higher torque for a stair walking, a larger motor and gear set should be applied, and the prosthetic leg must be relatively heavy due to their weight. The prosthetic leg structure was optimized with topology optimization to reduce its weight. Additionally, the ankle joint consists of a spring system to obtain a driving force to shift the body. The structure of the prosthetic leg was optimally designed with topology optimization to minimize weight while maintaining the safety of the structure. FE analysis was performed to verify the safety of the structure, and unlocked prosthetic leg test was carried out for testing the controller.

## 2. Design of the Motorized Prosthetic Leg System

### 2.1. Design Torque-Generating System

A transfemoral prosthetic leg is a rehabilitation apparatus for above-knee amputees. Thus, it is necessary for a prosthetic leg to implement the functions of the knee and ankle joints. Furthermore, it is necessary for a powered prosthetic leg to imitate the motion of each joint and to also possess dimensions similar to the body size to ensure user comfort. In this study, the walking mechanism and lower-limb structure were analyzed to determine the dimensions and performance of a prosthetic leg. A target user included a 28-year-old male with a body size involving a height of 176.6 cm and weight of 82 kg.

A previous study indicated that the specific weight of the shank and foot should correspond to 5.99% of the total body mass [18]. Therefore, the weight of the prosthetic leg should be less than 4.912 kg, which is set as the user's body weight. The length of the lower knee leg is measured for design.  Figure 1 shows portions of the lower knee leg segment in which the shank possesses a length of 37.3 cm from the knee to the ankle, and the foot is of the length of 6.5 cm. Based on a previous study, the highest knee torque of human gait occurs during stair descent, and the normalized value at that point is approximately 1.3 Nm/kg [19]. Given a user weight of approximately 82 kg, the knee joint of a prosthetic leg can produce a torque of up to approximately 106.6 Nm for functions similar to the human knee. Similarly, the highest plantarflexion moments of human gait occur during level walking, and the maximum normalized value was approximately 1.55 Nm/kg [19]. That is, the ankle joint could support a torque of 127.1 Nm.

The core of the prosthesis that can climb stairs should be light, creating a torque that is strong enough to support the human weight. When selecting torque, safety factor was considered excessively. Since the weight difference due to the reducer was not large compared to other parts, safety was prioritized over weight reduction of the motor within the range that satisfies the weight requirement.

Two types of torque generating systems exist at the knee joint, namely, the three linkage type and the direct-drive type. Conventional linkage types can easily convert linear motion to rotation motion, but the size cannot be reduced due to the geometry limitations. In this study, a BLDC (brushless DC) motor was used because the three linkage-type mechanism involves performance and weight limitations due to the dimensions of the linkage structure [20]. The concept model is shown in Figure 2. EC 45 BLDC motor made by Maxon (136211) was selected as the knee joint motor, given a maximum power production capacity of 250 W. The torque constant and nominal current of the motor corresponded to 0.0328 Nm/A and 10.2 A, respectively. If the maximum current was assumed as the nominal current, then the maximum torque of the motor corresponded to 0.3346 Nm. Therefore, a reduction gear with a gear ratio of 318.5 : 1 was used to achieve the maximum required torque of 106.6 Nm for the knee joint.

During stair walking, the specific aim was to control the joint angle along the reference motion. It was important to check motion stability, not to control in 0.1 degree units like a precision mechanical system. To confirm the feasibility of operation of the entire lightweight prosthetic system (3D printing structure), the experiment was conducted to see if the designed motorized prosthesis can properly follow the reference motion. It has been confirmed that the error of the angle and delay was shown at the degree level.

The spring system was introduced to create the required torque without the addition of a motor and electric devices at the ankle joint. The plate spring was used for the ankle joint because it was advantageous in terms of space applications. Additionally, FE analysis was used to determine the spring coefficient. The maximum required torque corresponded to 127.1 Nm, and the knee flexion angle at that point was approximately 15°. The geometrical relationship indicated that the displacement of the spring *δ* is based on the following equation: *δ* = *d*sin*θ*, in which *θ* = 15° and *d* = 35 mm. That is, the value of *δ* was approximately 9 mm. The thickness of the plate spring was determined by comparing the result of the FE analysis and the theoretical displacement *δ* at which they coincided.  Figure 3 shows the proper thickness of the plate spring calculated by FE analysis. The property of the spring was assumed as SAE1045, which is typically used for spring. This material possessed a density (*ρ*) of 7,700 kg/m^3^, elastic modulus (*E*) of 207 GPa, Poisson's ratio (*v*) of 0.266, and a yield stress of 1515 MPa. Finally, the proper thickness of the spring was determined, and the value corresponded to 0.5 mm.

The design specifications are summarized in Table 1. The design of the active transfemoral prosthetic leg utilizes the BLDC motor designed for the knee joint. A motor with planetary gear and helical bevel gear actuated the knee joint. The spring system generated torque for the driving force from the ground at the ankle joint. The knee joint was capable of 100° of flexion at the knee. Additionally, the ankle was capable of 25° of plantarflexion and 15° of dorsiflexion at the ankle.

### 2.2. Design Process and Topology Optimization

First, the specifications of the knee joint were defined to satisfy the reported boundary conditions for walking on stairs based on a previous study [19]. The major components, such as the motor and torque amplifier, were then determined. This was followed by designing a model and improving the model by topology optimization to reduce weight.

Topology optimization involves a mathematical method to obtain the optimal distribution of material for given design conditions including boundary conditions. The topology optimization problem was formulated in 1988 using a homogenization method [21]. Homogenization and solid isotropic material with penalization (SIMP) are widely used methods to solve optimization problems. These methods allow discrete design variables with intermediate density values ranging from 0 to 1. Specifically, SIMP is an extension of the homogenization method that has gained popularity in structural optimization because of its conceptual simplicity and ease of implementation [22].

Design variables, constraints, and an objective function are required to define an optimization problem. The problem for minimizing mass can be expressed as follows [23]:

Minimize: mass.

(1) $$\begin{array}{c} \text{Subject to }F\left(\sigma \left(x\right)\right)\leq 0,\forall \text{x}\in \Omega . \end{array}$$

The material failure function *F* depends on the stress field *σ*(*x*) and strain field *ε*(*x*), which are defined with respect to an original domain *Ω*. The failure function is defined with the von-Mises criterion, which is normally used as a failure criterion. The failure function *F* is expressed as follows:

(2) $$\begin{array}{c} F\left(\sigma \right)=\frac{\sigma_{v}}{\sigma_{e}}-1, \end{array}$$

where *σ*_*e*_ denotes the equivalent stress, which is usually regarded as the yield stress of the material, and *σ*_*v*_ denotes the effective von Mises stress that is computed as follows:

(3) $$\begin{array}{c} {\sigma_{v}}^{2}=\frac{1}{2}\left[{\left(\sigma_{11}-\sigma_{22}\right)}^{2}+{\left(\sigma_{22}-\sigma_{33}\right)}^{2}+{\left(\sigma_{33}-\sigma_{11}\right)}^{2}\right]+3\left({\sigma_{12}}^{2}+{\sigma_{23}}^{2}+{\sigma_{31}}^{2}\right). \end{array}$$

The density approach was used for topology optimization. The standard format of a linear static topology optimization problem is expressed as follows:

(4) $$\begin{array}{c} \mathrm{Minimize}:m=\overset{N.E.}{\underset{i=1}{\sum }}\rho_{i}\Omega_{i}\\ \text{Subject to F}\left(\sigma_{i}\right)\leq 0\\ \overset{N.E}{\underset{i=1}{\sum }}\rho_{i}V_{i}\leq V_{0}\\ 0<\rho_{\min}\leq \rho_{i}\leq 1 \end{array}$$

The number of elements in the design domain is denoted by N.E., and *Ω* represents the region occupied by a finite element. Furthermore, *V*_*O*_ denotes the volume of the design space, and it denotes the index of the elements. The design variable corresponds to the bulk material density, which can be expressed using relative material density and material properties of each element in the SIMP method. The elasticity tensor (*E*) includes the following relationship:

(5) $$\begin{array}{c} E\left(\rho \right)=\rho^{n}E_{0}, \end{array}$$

where *n* denotes a penalization factor, and *ρ* denotes the density (0 ≤ *n*, 0 ≤ *ρ* ≤ 1) [20, 24].

The optimization process and particularly topology optimization converge during the process of developing an active transfemoral prosthetic leg.

The objective of optimization involved determining the optimized structure while ensuring structural safety under working conditions. There are three design optimization methods, namely, shape optimization, size optimization, and topology optimization. Shape optimization involves determining the optimum shape by adjusting the positions of each node on the outer surface of the structure under boundary conditions. Size optimization involves a process of determining the properties of structural elements such as shell thickness, beam cross-sectional properties, spring stiffness, and mass. Finally, topology optimization involves finding an optimized structure by utilizing internal strain energy density distributions and removing any portion that does not contribute to the structural strength. These optimization processes were applied to design the structure of an active transfemoral prosthetic leg.

Additionally, NX 9.0 was used for 3D CAD modeling. Shape optimization was implemented by Optistruct Solver of Altair Hyperworks, and Inspire of SolidThinking was used as the solver for topology optimization. The optimization process commenced with the definition of the design space. It was necessary to maximize the design space while minimizing the space for other components and interference caused by the rotating motion of joints. The nondesign space, such as connections to bearings and bolts, in which optimization is not performed, was defined. The FE model was introduced for optimization, and properties of the material and the boundary conditions including external load were applied. The design parameters for optimization were set and included design variables, objective function, constraints, and the minimum or maximum size of the structure. Following the preprocessing, an optimization process was performed to determine the optimal structure while satisfying the constraints. This was followed by performing optimization with iterations until the performances satisfied the objective function. After the optimization process, the optimized shape was designed given the optimization results. Finally, the optimized model was verified by FE analysis.

### 2.3. Structural Design of Artificial Foot

A prosthetic foot includes malleability to accommodate variation in the physical terrain in conjunction with rigidity to enable transmission of the body weight with adequate stability [25]. Therefore, plastic nylon was used to develop the artificial foot because it possesses sufficient flexibility to absorb shocks while supporting the body weight. It is necessary for the artificial leg to look similar to a human foot because several amputees desire to be perceived as normal. Therefore, it is important that the shape of the artificial foot is similar to that of a human foot and for the size to not exceed real foot size.

A few conditions involving the peak ground reactant force were considered to design the foot structure. According to the previous study [19], the peak ground reaction force appeared during stair descent walking with a magnitude that corresponded to 1.5 times the body weight of a human. The maximum ankle moment corresponded to 1.55 Nm/kg and occurred at the end of the stance phase and was also considered as a boundary condition. Additionally, the anterior/posterior ground reaction force was also considered as a boundary condition. Two notable points occurred at 20% and 85% of the stance phase of level walking. One of the points involved the heel-strike phase in which the magnitude corresponded to 0.15 times the body weight, and the other point involved the toe-off phase in which the magnitude corresponded to 0.2 times the body weight. The peak values at these points were considered as a boundary condition. The medial/lateral ground reaction force is relatively small and is therefore negligible. The boundary conditions for optimization were determined considering the abovementioned walking characteristics and are shown in Figure 4. There are three load cases for the boundary condition, and optimization was performed by simultaneously applying all three cases as each case was considered independent. The load was imposed on the ankle joint, and fixed boundary conditions were applied to the ball of the foot and heel that were directly in contact with the ground. The foot material corresponded to plastic nylon, which possessed flexibility and robustness. The material had a density (*ρ*) of 1,230 kg/m^3^, an elastic modulus (*E*) of 2.91 GPa, a Poisson's ratio (*v*) of 0.41, and an yield stress of 75 MPa.

Following the definition of the boundary condition and materials, topology optimization was performed to design the optimal shape of the structure.  Figure 5(a) shows the maximum designable space, which was maximized while avoiding the space for other components and interference caused by the rotating motion of the ankle joint. The nondesign space where optimization was not performed was defined at the contact surface and joint. The design space was used for topology optimization using boundary conditions, as shown in Figure 4 and applying a material corresponding to plastic nylon.  Figure 5(b) shows the topology optimization results. The unnecessary mass was eliminated while maintaining the robustness under the boundary condition. However, it was too complicated to directly manufacture the shape by machining, and thus, 3D printing was used to realize the model. 3D printing is advantageous as it can create complicated shapes. Therefore, the result of optimization can be applied in a very similar manner by using 3D printing.  Figure 5(c) shows the optimized model that was designed based on the topology optimization results and manufacturing method. Finally, the optimized foot was manufactured by a 3D printer and is shown in Figure 5(d).

### 2.4. Structural Design of the Lower Limb

It is necessary for the lower-limb structure of a prosthetic leg to sustain the body weight of the user and bear an approximate torque of 106.6 Nm for the same function as the human knee when a user's weight corresponds to 82 kg. The body weight is assumed as the maximum ground reaction force, which corresponds to 1205.4 N. A previous study [26] indicated that the resultant ground reaction forces were directed towards the center of gravity. Therefore, the resultant force of the ground reaction forces was assumed to be in the same direction as the shin. Additionally, the torque imposed on the knee joint was supported by the structure of the lower limb and the gear system. Constraints were applied at the end of the bottom of the prosthetic leg, which was connected to an adapter and was assumed as a fixed joint. The boundary condition for optimization was determined considering the abovementioned load conditions and is shown in Figure 6.

It is necessary for the material of the lower-limb structure to exhibit robustness for safety and ensuring weight lightness with respect to user comfort. Thus, 7075 aluminum alloy was used as the design material for the lower-limb structure. This material is usually used for prostheses and is lighter than steel alloy. This material includes a density (*ρ*) of 2,800 kg/m^3^, an elastic modulus (*E*) of 75 GPa, a Poisson's ratio (*v*) of 0.33, and a yield stress of 95 MPa.

Similar to the structural design, the optimization process was implemented to design the optimal structure by considering boundary conditions.  Figure 7(a) shows the maximum designable space for the lower-limb structure. It was necessary for the maximum designable space to not exceed the dimensions of a human leg and to avoid interferences with other components such as motors and gearbox. The bearings and bolts defined the nondesign space in which optimization was not performed. The design space was used for topology optimization using boundary conditions based on Figure 8 and an aluminum alloy.  Figure 7(b) shows the topology optimization results. In this phase, geometrical symmetry was considered for the balance of the prosthesis. The result indicated that the shape of the structure did not significantly differ from that of the previous model despite changes in the thickness and edge. Following the topology optimization, shape optimization was implemented to obtain a better model by determining the thickness as shown in Figure 7(c). The degree of freedom of nodes placed on the outer face of the upper structure and the inner face of the lower structure were considered as a design variable. The constraints and external force were the same as the boundary conditions for topology optimization. The objective function involved minimizing the mass. The contour showed the displacement of the shape change versus the original model. The results indicated that it was necessary to reduce the thickness to approximately 6 mm. The optimal thickness of the structure was determined based on the results. Finally, the advanced shape of the lower-limb structure was obtained while maintaining robustness under boundary conditions. Figures 7(d) and 8(d) show 3D modeling and the model manufactured by machining, respectively.

### 2.5. Design of the PD Controller

An important point in the development of active transfemoral prosthetic leg involves implementing the motion of natural gait using a power source. It is important to analyze human gait to determine the walking phase and to implement the motion of the affected side that is similar to that of the normal side. In this study, a walking phase was identified through a mechanical sensor for knee joint control, and the PD controller based on the knee angle position was applied to actively cope with various walking environments.

An encoder was used to collect the walking motion data of the knee joint to analyze the walking behavior. The measuring system is shown in Figure 9. The gait data of each walking situation were collected by walking around stairs and flat ground. The data were measured five times for each case. The noise was removed by filtering, and the standard gait data was determined by averaging. The data of a level and the stair walking are shown in Figure 10, and this was used as a trajectory to implement the walking motion.

The swing motion was implemented by entering the motion to track on the motor for tracking obtained from Figure 10. The dynamic relationship of the walking system is as follows [23]:

(6) $$\begin{array}{c} \tau =k\left(\theta -\theta_{\text{eq}}\right)+b\dot{\theta }, \end{array}$$

where *τ* denotes the torque of the knee and ankle joint, and *k* and *b* denote the linear stiffness and damping coefficient, respectively. Additionally, *θ* denotes the angle of the knee joint, and *θ*_eq_ denotes the equilibrium angle during the transition between phases. A position-based PD controller was constructed to control the active prosthetic leg and applied to the developed prosthesis. Based on previous studies, the parameters were tuned using a combination of feedback from the user and from visual inspection of the joint angle, torque, and power data [27].

In the PD controller, a control loop feedback mechanism that is commonly used in industrial control systems is used for control. The control system is shown in Figure 11. The PD controller is used to mitigate the stability and overshoot problems that arise when a proportional controller is used at a high gain by adding a term proportional to the time derivative of the error signal. The value of the damping can be adjusted to achieve a critically damped response.

The decomposition of the joint behavior into passive segments requires division of the gait cycle into modes or “finite states” [8]. The walking phase was distinguished by the load cell and the encoder signal. A finite state machine was constructed as shown in Figure 12 to further divide the walking step into four steps. The finite state machine of the prosthetic leg was based on previous studies [9, 27, 28].

Phase 1 constitutes the stance phase. If the knee was extended over a certain angle in swing flexion, then the phase switched to the stance phase. The sole had contact with the ground, and the load was applied to the knee joint. If the heel strike or forefoot strike was detected through the load cell attached to the middle of the structure, then the walking phase was changed from the prelanding phase to the stance phase.

Phase 2 constitutes the preswing phase. This phase immediately preceded the detachment of the sole from the ground, and the load on the knee moved to the opposite leg. The heel fell from the ground while the knee bent over a certain angle, and this was followed by changing the walking phase into the preswing phase.

Phase 3 constitutes the swing flexion phase. When the sole was completely separated from the ground, the load on the knee was completely free because the load was supported by another side leg. When the load cell confirmed that the foot was completely separated from the ground, the walking phase changed from the preswing phase to the swing flexion phase.

Phase 4 constitutes the swing extension phase. The knee joint began to naturally expand. If the direction of the angular velocity of the knee joint was reversed in the swing flexion phase, then the walking phase changed into the swing extension phase.

An experimental method was used to perform coefficient adjustment of the controller to optimize the walking performance of the active prosthesis system.

## 3. Validation of the Developed Prosthetic Leg

### 3.1. Artificial Foot Structure Analysis

It is necessary for the artificial foot to support body weight while walking. Therefore, FE analysis was performed to validate its structural safety. The abovementioned boundary condition was applied. FE analysis was performed for each of the boundary conditions.  Figure 13 shows the 3D mesh and boundary conditions for the analysis. The quality of the mesh was important for obtaining an accurate result. A tetra mesh was used due to its advantages in meshing a complex solid shape. The outer surfaces and geometrical corners involved compact meshes for accurate analysis. The number of elements corresponded to 141,898, and the number of nodes corresponded to 38,047. The model included three load cases consisting of heel strike, toe off, and mid-stance. The external loads and moment of each load case acted on the center of the ankle joint, and constraints were applied to the ball of the foot and heel. All the materials were modeled as linearly elastic, isotropic, and homogenous.  Figure 14 shows the results of the FE analysis of the foot structure.  Table 2 summarizes the peak stresses of each phase. The highest von Mises stresses appeared in the heel strike phase, which was located at the lower surface of the heel. The maximum stress obtained in the results was compared with the tensile strength of the materials used to check the stability with respect to the applied load. The maximum stress corresponded to 65.51 MPa, which was lower than the yield strength of the material (75 MPa).

### 3.2. Lower-Limb Structure Analysis

In order to verify the safety of the structure, FE analysis was performed under a boundary condition similar to that shown in Figure 6.  Figure 15(a) shows the 3D mesh for the analysis. A tetra mesh was used owing to its advantages in meshing a complex solid shape. The number of elements corresponded to 365,724, and the number of nodes corresponded to 84,988.

The body weight was applied to the nodes located at the center of the bearing holes that supported the knee shaft. The twelve bolt connections between the support and bevel gearbox were considered as rigid link components based on the assumption that the bolts were nearly rigid bodies with little deformation. Fixed constraints were applied to the bolt hole located at the bottom of the leg that was bolted with a pyramid adaptor. All the materials were modeled as linearly elastic, isotropic, and homogenous.

The results of the FE analysis of the lower-limb structure are shown in Figure 15(b). The maximum stress was exhibited in the area near the bolt hole. The value was 80.71 MPa lower than 95 MPa, which corresponded to the yield strength of the 7075 aluminum alloy. This implied that the structure was safe under the load condition. Furthermore, the bolt holes were simplified to a rigid element, and it displayed a characteristic indicating a stress that exceeded the real stress because the rigid element acted as a load point. Therefore, it was expected that the actual stress at the point was lower than 80.71 MPa.

### 3.3. Unlocked Prosthetic Leg Test

An experimental setup for the unlocked prosthetic leg test was introduced to create the motion of the knee joint. The experimental setup is shown in Figure 16, and it was designed to ensure that the prosthetic leg could move freely. The coefficient adjustment of the controller to optimize the walking performance of the active prosthesis system was performed through an experimental method. Given the reference walking data and user feedback, the value that could mimic the walking motion in the most natural manner possible was selected as the coefficient value. Tables 3, 4, and 5 show the coefficient of the controller for level walking, stair ascent, and descent, respectively. The controller coefficients for each phase were obtained through the experimental method. The equilibrium angle *θ*_eq_ was selected as the peak angle of each phase or the angle at which the ground reaction force was imposed.

## 4. Discussion

### 4.1. Performance Evaluation of Prosthetic Leg

Consequently, an active transfemoral prosthetic leg system was developed as shown in Figure 8. The three linkage type includes certain specification disadvantages, and thus, a direct-drive type was applied to the knee joint, and a spring system was applied to the ankle joint. The structure was then designed using the optimization process. The active prosthesis was designed with two degrees of freedom in the ankle and knee. The knee joint plays an important role and is accountable for more than 50% of the walking mechanism. It consists of an AC motor system and can generate 106.57 Nm torque and proper motion in a range from 0° to 100°. The ankle joint plays an important role in supporting the torque caused by the body weight. The spring system is simple and involves a general system to generate torque without a motor system. The ankle joint was composed of a spring system to generate 127.1 Nm torque and angle.

In order to evaluate design efficiency, specifications of the prosthetic leg system and desired specifications were compared, and the comparison results are shown in Table 6. The objects of comparison included the maximum torque and operating angle of each joint, power of the knee joint, height, total weight, and maximum stress. These variables were selected for the following reasons.

First, it is necessary for the prosthetic leg to make a proper motion to mimic the gait of a normal person. Therefore, it is necessary for the prosthetic leg to implement the range of motions similar to a human leg in conjunction with supplying the necessary power to overcome obstacles that could be encountered by the amputees while walking. The range of the joint angle, target torques, and power was based on specifications listed in a previous study. The prosthetic leg was designed to meet the specification based on this design parameter.

Second, weight is the most important factor because the user can feel fatigue or discomfort if the prosthetic leg is heavier than their original leg. Hence, it is necessary to minimize the weight to ensure the comfort of the amputees. The developed active transfemoral prosthetic leg has a total weight of 4,779 g, which corresponds to 97.3% of the target weight (4,912 g) obtained by considering the user's body size. The weight of the prosthesis is 1.150 kg for the motor, 0.920 kg for the reducer, 0.209 kg for the foot, and 2.5 kg for the body (including cover and joint gear), totaling 4.779 kg. In addition, the experiment was conducted by supplying power by wire without a battery. Although the weight of the motor and gearbox exceeds 2 kgf, the total weight was effectively reduced by introducing an optimization process with respect to the structure. Similarly, it was necessary for the total length of the prosthetic leg to be similar to the length of the original leg of a user. The developed prosthetic leg had a length of 444.5 mm, which corresponded to 101.5% of the target length (438 mm).

Finally, it was necessary to ensure the safety of the user while using the prosthetic leg. Therefore, the safety factor is important in designing a prosthetic leg. The yield stress of the used material was compared with the maximum stress predicted by FE analysis. Plastic nylon (which is the foot structure material) has a yield strength of 75 MPa. The maximum stress of the foot structure was expected as 65.51 MPa, and the safety factor at this time was estimated as 1.15. In a similar manner, the 7075 aluminum alloy, which was used to design the material of the lower-limb structure, possesses a yield strength of 95 MPa. The maximum stress of the lower limb was expected as 80.71 MPa, and the safety factor at this time was estimated as 1.18. The maximum stresses of each part were lower than the yield strength of each material.

The developed prosthesis was heavier than the prosthesis sold on the market, although it was lighter than the dimensions of an actual human body. The weight of the motor and the gearbox exceeded 2 kg. It was necessary to introduce a suitable motor and gearbox to reduce the weight. Hence, the implementation of the research on optimizing motors and gearboxes will help in developing a better prosthesis.

### 4.2. Performance Evaluation of Controller

The comparison between the desired motion and the actual drive motion with the level walking controller obtained by the unlocked prosthetic leg test (Figure 17(a)). The knee angle of the prosthesis was measured while tracking the normal walking data. The actual motion of the prosthetic knee joint exhibited a similar tendency with the desired motion. The knee angle of the prosthetic leg indicated a smooth swing curve, but was relatively smaller than the desired angle and experienced a slight delay. This phenomenon was due to the limitations of the experimental system. The supplied voltage was lower than the nominal voltage and reduced the torque below the target torque. It was considered that the torque estimated by the influence of relatively low power supply had a slight delay when compared to the objective data and would thereby affect the walking speed.

Figures 17(b) and 17(c) show the comparison between the desired motion and the actual drive motion with stair ascent and the descent controller obtained by the unlocked prosthetic leg test. They also indicated that the objective function was followed in a similar manner. However, they exhibited slight inconsistencies. It involved a position-based control, and a delay occurred when each phase went to the next phase. This appeared to be the cause of showing the actual knee motion follow slightly refracted curves.

The active prosthetic leg and controller exhibited behavior that was considerably similar to that of a normal gait. The PD controller implemented a knee motion similar to normal walking. The experimental result of control based on the position data showed the feasibility of the level and stair walking of the active prosthetic leg using the PD controller. Additionally, it allowed the framework of the walking test to mimic the motion of a normal individual.

Finally, the developed prosthetic leg was controlled by a PD controller that generated human-like walking motion, and the resulting joint kinematics were compared with a captured human gait to verify the control performance. It is expected that the study results with respect to the active transfemoral prosthetic leg will help in the rehabilitation of amputees. Furthermore, this study can be applied to the area of biped robots that imitate the human motion.

## 5. Conclusions

In this study, an active transfemoral prosthetic leg was optimally designed and controlled with a PD controller. The weight of the prosthetic leg is an important factor in the design because it is related to user fatigue. An optimization process was used for foot and lower-limb structures to obtain optimal shapes and reduce the weight. Topology and shape optimization were implemented in the design. As a result, the shape of a prosthetic leg was developed without exceeding the dimensions of the human body. The optimized foot structure was produced through 3D printing to reflect the optimization result as much as possible. Finally, an optimized structure for stair walking was designed while maintaining robustness. A PD controller based on position control was used to control the developed prosthetic leg. The actual motion of the prosthetic knee joint exhibited a tendency similar to the desired motion. It is expected that the results of this study will aid in the rehabilitation of amputees by developing optimal active transfemoral prosthetic legs. Furthermore, the findings of this study can be applied to the area of biped robots wherein human motion is imitated.

## Figures and Tables

**Figure 1:** Dimensions of the lower knee leg.

**Figure 2:** Concept modeling of a powered transfemoral prosthetic leg.

**Figure 3:** FE analysis to obtain the proper thickness of the plate spring at the ankle joint.

**Figure 4:** Boundary conditions for foot optimization.

**Figure 5:** Optimization process for the foot structure.

**Figure 6:** Boundary conditions for lower-limb optimization.

**Figure 7:** Optimization process for lower-limb optimization.

**Figure 8:** Developed active prosthetic leg system.

**Figure 9:** Measuring system of the knee motion.

**Figure 10:** Measuring result of the knee motion.

**Figure 11:** PD controller for the knee motion control.

**Figure 12:** Finite state machine.

**Figure 13:** A 3D mesh of the foot structure and the boundary conditions.

**Figure 14:** Results of the FE analysis of the foot structure.

**Figure 15:** Result of the FE analysis of the lower-limb structure.

**Figure 16:** Experimental setup for the unlocked prosthetic leg test.

**Figure 17:** Comparison between the desired motion and the actual drive motion.

**Table 1:** Design objectives considering body dimensions.

Specification	Value
Knee range of motion	0° to 100°
Ankle range of motion	−25° to 15°
Maximum knee torque	106.6 nm
Maximum ankle torque	127.1 nm
Peak knee power	250 W
Height (below knee)	438 mm
Maximum total weight	4.912 kg

**Table 2:** Peak stresses of each walking phase.

Walking phase	Max stress	Yield stress
(a) Heel strike	65.51 MPa	75 MPa
(b) Toe off	64.56 MPa	
(c) Mid-stance	49.29 MPa	

**Table 3:** Coefficient of controller for level walking.

Phase	*k* (nm/deg)	*b* (ns/m)	*θ*eq (deg)
1	6	0	25
2	4	0	13
3	0.1	0.02	59
4	0.2	0.03	9

**Table 4:** Coefficient of controller for stair ascent.

Phase	*k* (nm/deg)	*b* (ns/m)	*θ*eq (deg)
1	2	0	17
2	10	0	24
3	0.1	0.02	87
4	0.5	0.03	72

**Table 5:** Coefficient of controller for stair descent.

Phase	*k* (nm/deg)	*b* (ns/m)	*θ*eq (deg)
1	8	0	28
2	6.5	0	26
3	0.1	0.02	81
4	0.1	0.03	13

**Table 6:** Comparison between the desired and prosthetic leg specifications.

	Requirement	Prosthetic leg
		Specifications
Knee range of motion	0° to 100°	0° to 100°
Ankle range of motion	−25° to 15°	−25° to 15°
Maximum knee torque	106.6 nm	106.57 nm
Maximum ankle torque	127.1 nm	127.1 nm
Peak knee power	250 W	250 W
Height (below-knee)	438 mm	444.5 mm
Maximum total weight	4.912 kg	4.779 kg
Max. stress	Foot: 65.51/75 MPa	
Allowable stress	Lower limb: 80.71/95 MPa	

## Data Availability

The experimental and simulation data used in this study are included within the paper.

## References

[1] Sup F., Varol H. A., Mitchell J., Withrow T. J., Goldfarb M. Self-contained powered knee and ankle prosthesis: initial evaluation on a transfemoral amputee.

[2] Martinez-Villalpando E. C., Herr H. (2009). Agonist-antagonist active knee prosthesis: a preliminary study in level-ground walking. *Journal of Rehabilitation Research & Development*.

[3] Russell Esposito E., Aldridge Whitehead J. M., Wilken J. M. (2016). Step-to-step transition work during level and inclined walking using passive and powered ankle–foot prostheses. *Prosthetics and Orthotics International*.

[4] Realmuto J., Klute G., Devasia S. (2015). Nonlinear passive cam-based springs for ankle prostheses. *Journal of Mecial Devices*.

[5] Sup F., Varol H. A., Goldfarb M. (2011). Upslope walking with a powered knee and ankle prosthesis: initial results with an amputee subject. *IEEE Transactions on Neural Systems and Rehabilitation*.

[6] Flowers W. C., Mann R. W. (1977). An electrohydraulic knee-torque controller for a prosthesis simulator. *ASME Journal of Biomechanical Engineering*.

[7] Lee K. H., Chung J. H., Lee C. H. (2013). Design and optimization study of active trasfemoral prosthesis leg. *Korean Journal of Rehabilitation Welfare Engineering & Assistive Technology*.

[8] Sup F., Bohara A., Goldfarb M. (2008). Design and control of a powered transfemoral prosthesis. *The International journal of robotics Research*.

[9] Lawson B., Varol H. A., Huff A., Erdemir E., Goldfarb M. (2013). Control of stair ascent and descent with a powered transfemoral prosthesis. *IEEE Transactions on Neural Systems and Rehabilitation Engineering*.

[10] Au S., Berniker M., Herr H. (2008). Powered ankle-foot prosthesis to assist level-ground and stair-descent gaits. *neural networks*.

[11] Grimmer M. (2016). A powered prosthetic ankle joint for walking and running. *Biomedical Engineering*.

[12] Yang U. J., Kim J. Y. (2015). Mechanical design of powered prosthetic leg and walking pattern generation based on motion capture data. *Advanced Robotics*.

[13] Bellman R. D., Holgate M., Sugar T. G. Design of an Active Robotic Ankle Prosthesis with Two Actuated Degrees of Freedom Using Regenerative Kinetics.

[14] Borjian R., Lim J., Khamesee M. B., Melek W. The design of an intelligent mechanical active prosthetic knee.

[15] Ha K. H., Varol H. A., Goldfarb M. (2011). Volitional control of a prosthetic knee using surface electromyography. *IEEE Transactions on Biomedical Engineering*.

[16] Bernal-Torres M. G., Medellin-Castillo H. I., Arellano-Gonzalez J. C. (2018). Design and control of a new biomimetic transfemoral knee prosthesis using an echo-control scheme. *Journal of Healthcare Engineering*.

[17] Omasta M., Paloušek D., Návrat T., Rosický J. (2012). Finite element analysis for the evaluation of the structural behaviour, of a prosthesis for trans-tibial amputees. *Medical Engineering & Physics*.

[18] Ho W. H., Shiang T.-Y., Lee C. C., Cheng S. Y. (2013). Body segment parameters of young Chinese men determined with magnetic resonance imaging. *Medicine & Science in Sports & Exercise*.

[19] Riener R., Rabuffetti M., Frigo C. (2002). Stair ascent and descent at different inclinations. *Gait & Posture*.

[20] Lee K. H., Chung J. H., Lee C. H. Development of artificial foot of active transfemoral prosthesis system using topology optimization.

[21] Bendsøe M. P., Kikuchi N. (1988). Generating optimal topologies in structural design using a homogenization method. *Computer Methods in Applied Mechanics and Engineering*.

[22] Luo Z., Zhang N., Wang Y., Gao W. (2012). Topology optimization of structures using meshless density variable approximants. *International Journal for Numerical Methods in Engineering*.

[23] Pereira J. T., Fancello E. A., Barcellos C. S. (2004). Topology optimization of continuum structures with material failure constraints. *Structural and Multidisciplinary Optimization*.

[24] Cha S. H., Lee S. W., Cho S. (2013). Experimental validation of topology design optimization. *Computational Structural Engineering Institute of Korea*.

[25] Saunders M. M., Schwentker E. P., Kay D. B. (2003). Finite element analysis as a tool for parametric prosthetic foot design and evaluation. Technique development in the solid ankle cushioned heel (SACH) foot. *Computer Methods in Biomechanics and Biomedical Engineering*.

[26] Levine D., Richards J., Whittle M. W. (2012). *Whittle's gait analysis*.

[27] Sup F., Varol H. A., Mitchell J., Withrow T. J., Goldfarb M. (2009). Preliminary evaluations of a self-contained anthropomorphic transfemoral prosthesis. *IEEE/ASME Transactions on Mechatronics*.

[28] Kim W. S., Kim S. Y., Lee Y. S. Prototype development of a DC motor-based powered prosthesis and its control.

